The article "Novel Method of Analysis for the Determination of Residual Formaldehyde by High-Performance Liquid Chromatography" was published in 2022. Journal: Int J Anal Chem.

# Novel Method of Analysis for the Determination of Residual Formaldehyde by High-Performance Liquid Chromatography

**DOI:** 10.1155/2022/9171836

**Published:** 2022-09-06

**Authors:** Vittoria Delbono, Christopher P. Larch, Katrina Carol Newlands, Shona Rhydderch, Thomas Craven Baddeley, John Mervyn David Storey

**Affiliations:** ^1^Department of Chemistry, School of Natural and Computing Sciences, University of Aberdeen, Aberdeen AB24 3UE, UK; ^2^TauRx Therapeutics Ltd, 395 King Street, Aberdeen AB24 5RP, UK

## Abstract

Formaldehyde is commonly used as an alkylating agent in the pharmaceutical industry. Consequently, its residual level in drug substances and/or their intermediates needs to be accurately quantified. Formaldehyde is a small, volatile molecule with a weak chromophore (the carbonyl group), and its direct analysis by GC-FID and HPLC-UV is difficult. For these reasons, the majority of papers found in the literature are based upon a derivatisation process (most commonly using the desensitised explosive 2,4-dinitrophenylhydrazine) prior to the analysis of formaldehyde. A novel high-performance liquid chromatography (HPLC) method with UV detection for its quantification in a pharmaceutical is described in this paper. The method proposed herein is based upon a derivatisation reaction between formaldehyde and 4-methylbenzenesulfonohydrazide (MBSH) before analysis by HPLC-UV. Selectivity, linearity, limit of quantification, accuracy, repeatability, intermediate precision, and solution stability were successfully assessed as per ICH guideline Q2(R1), and the method has also been validated in a good manufacturing practice (GMP) laboratory in the UK.

## 1. Introduction

Formaldehyde is a naturally occurring, colourless gas to which people are exposed to daily. It is present in the environment as a result of natural processes (e.g., in photochemical and metabolic processes in plants, animals, and humans) and from man-made sources, with incomplete combustion of hydrocarbons being the major source of atmospheric formaldehyde [1, 2]. Formaldehyde is also prevalent at quite high levels in some food, such as fruit and marine fish [1, 2]. Frequently higher levels of formaldehyde are present indoors compared with outdoors due to its presence in paints, varnishes, and several synthetic wood products [2].

The toxicity of formaldehyde has been extensively investigated during the last decades [1–5] and was found to cause both acute and chronic effects in humans, particularly through inhalation, causing irritation to the eyes, nose, and throat [2]. Despite its toxicity, formaldehyde is essential for several biochemical pathways in humans (e.g., lipid metabolism in the decomposition of peroxides by catalase [5]) with endogenous formaldehyde being measured in the body at concentrations of approximately 100 *μ*M [3].

The article "Novel Method of Analysis for the Determination of Residual Formaldehyde by High-Performance Liquid Chromatography" was published in 2022. Journal: Int J Anal Chem.

Formaldehyde is a valuable alkylating agent used in the industrial manufacture of pharmaceuticals, and it can be employed in solution form (i.e., formalin) or in polymeric form (e.g., paraformaldehyde). Regulatory guidelines for manufacturing and marketing require that formaldehyde concentrations are strictly monitored in these products [6, 7]. Therefore, methods to quantify formaldehyde with high sensitivity and accuracy are of considerable importance and interest.

Unfortunately, formaldehyde has a weak chromophore and its direct analysis by commonly used detectors in the pharmaceutical industry (i.e., flame ionisation and UV) is difficult. For these reasons, previously published methods for its quantification are predominantly based upon a derivatisation process prior to analysis.

Formaldehyde analysis has been extensively studied for many years. Analytical methods have been developed to determine formaldehyde in numerous matrices, such as cosmetics, food, drink, environmental samples, and pharmaceuticals. These methods are based on various analytical techniques, such as high-performance liquid chromatography ultraviolet detection (HPLC-UV) [8–14], gas chromatography flame ionisation detection (GC-FID) [15, 16], mass spectrometry [17–19], fluorescence [20–23], spectrophotometry [24, 25], chromotropic acid spectrophotometry [26], photoluminescence [27], and capillary electrophoresis [28]. Sensors and probes for formaldehyde have also been explored [29–33].

Fluorescence derivatisation methods [20–23] are based upon reactions forming compounds possessing fluorescence properties. These include reaction of aldehydes with *β*-diketones (Hantzsch reaction), such as 2,4-pentanedione [34] and 1,3-cyclohexanedione [35], Fluoral-P [36–39], anthrone [40], m-aminophenol [41], and ampicillin [21], with the latter showing lack of selectivity [42]. Applications to aquatic products, biological samples, packaging paper, food, alcoholic beverages, alcohol fuels, and air samples have been reported. Although it could potentially be applied to pharmaceutical samples too, this detection technique, as well as photoluminescence and capillary electrophoresis, is not yet widely available across testing laboratories for this type of samples. Also, probes can be good alternatives for their simplicity, high sensitivity, rapidity, ease of application, and real-time monitoring, but their application has been to date been limited to specific matrices, such as living cells, tissues, and environmental samples.

Spectrophotometric methods may represent an appropriate low cost alternative to chromatographic methods, but these generally present spectral interferences, therefore showing poor selectivity, and they can lack sensitivity.

The article "Novel Method of Analysis for the Determination of Residual Formaldehyde by High-Performance Liquid Chromatography" was published in 2022. Journal: Int J Anal Chem.

For the purpose of this work, special attention was given to HPLC and GC methods, as these techniques are more widely used within the pharmaceutical industry for routine use.

Hu et al. [15] proposed a method in which formaldehyde is reduced to methanol and subsequently analysed by GC-FID. However, methanol demonstrates a poor response by FID, compromising the sensitivity of the method. Furthermore, the basic pH of the diluent used limits this method to samples that are stable in basic conditions; otherwise, unpredictable decomposition may well interfere with the analysis. The same drawback has been encountered for the derivatisation using acetylacetone and ammonia [9], pentafluorobenzyl hydroxylamine [19], and ethyl 3-oxobutanoate and ammonia [8].

Sensitive methods can be achieved through derivatisation and successive analysis by mass spectrometry detectors, as reported by Li et al. [17] and del Barrio et al. [18]; however, mass spectrometers are not common in laboratories that conduct routine Active Pharmaceutical Ingredient (API) testing, so, while suitable for larger organisations and research environments, other methods are still sought.

Other derivatisation processes have also been reported [16, 43], with the use of 2,4-dinitrophenylhydrazine (DNPH) being the most widely cited technique, usually followed by analysis by HPLC-UV [11–14, 44–57]. However, due to the explosive nature of DNPH and its reactivity towards oxidising reagents, commercially available DNPH in powder form contains at least 33% of water and this water content can be variable and change over time necessitating strict precautions for its storage as it can ignite if allowed to dry. This led to the need of safely disposing of this material by competent personnel in many schools around the UK back in 2016–2017 [58–62]. For these reasons, DNPH transportation by aircraft is also not permitted. Furthermore, the need for the compound to contain high water content (not less than 30%) leads to high volumes being transported and the necessity to determine the water content prior to use presenting its own operational difficulties. In this paper, we wish to detail the development of an alternative robust method that can be used to accurately quantify formaldehyde found in pharmaceuticals and pharmaceutical intermediates, employing an alternative derivatising reagent, which is safer to store and transport than solid DNPH. Such a development is particularly important when methods need to be reproduced worldwide in different contract manufacturing organisations (CMOs).

The article "Novel Method of Analysis for the Determination of Residual Formaldehyde by High-Performance Liquid Chromatography" was published in 2022. Journal: Int J Anal Chem.

Consequently, an alternative method for the selective analysis of formaldehyde in base-sensitive samples using a widely accessible and safer derivatising reagent for storage and transportation and a widespread technique of analysis in the pharmaceutical industry (HPLC-UV) was pursued.

The method proposed herein is based upon a reaction between formaldehyde and 4-methylbenzenesulfonohydrazide (MBSH) and subsequent analysis by HPLC-UV. The resulting formaldehyde/MBSH derivative, postulated in Figure 1, possesses a strong chromophore, thus enabling detection by the mentioned technique.

The formation of the target imine starts with the nucleophilic attack on the carbonyl of formaldehyde by the primary amine of MBSH in the presence of acetic acid. This reaction is concerted due to the unstable carbinolamine intermediate. The resulting 1-(hydroxymethyl)-2-(4-methylbenzene-1-sulfonyl)hydrazin-1-ium intermediate loses one unit of water, facilitated by acetic acid, which results in the formation of the formaldehyde/MBSH derivative, 4-methyl-*N*′-methylidenebenzene-1-sulfonohydrazide.

## 2. Materials and Methods

### 2.1. Chemicals and Materials

Acetonitrile (HPLC grade), p-toluene sulfonyl hydrazide (4-methylbenzenesulfonohydrazide/MBSH, 97%), acetic acid (100%), and formaldehyde (37% w/v in water, containing 10–15% methanol) were all purchased from Merck KGaA (Darmstadt, Germany). Formic acid (99–100%) was purchased from VWR (Radnor, Pennsylvania, USA). The UHQ water (≤18 MΩ) was supplied in house by a Milli-Q direct 8 water purification system (Millipore, Burlington, Massachusetts, USA).

A MBSH solution in acetonitrile (2 mg/mL) was prepared by dissolving 100 mg of MBSH in acetonitrile to a volume of 50 mL. An acetic acid solution (200 *μ*g/mL) was prepared by dissolving 10 *μ*L of acetic acid in 50 mL of water. Methylthioninium chloride (MTC) samples 1–6 were provided by TauRx Therapeutics Ltd (Aberdeen, United Kingdom).

### 2.2. Standard and Sample Preparation

A formaldehyde stock solution (500 *μ*g/mL) was prepared by diluting the 37% (w/v) formaldehyde solution with water. This solution was further diluted with water to solutions of 0.5, 1.0, 2.5, 5.0, 10.0, and 15.0 *μ*g/mL formaldehyde (corresponding to 83, 167, 417, 833, 1250, 1667, and 2500 *μ*g/g in the material) for the calibration curve and of 6.0 *μ*g/mL for standard accuracy and repeatability testing. Into a suitable vial, 5.0 mL of each standard solution was added. Samples were weighed (30 mg) into a suitable vial, followed by the addition of 5.0 mL of water. Sonication was applied for about 10 minutes to ensure complete dissolution of the sample.

The article "Novel Method of Analysis for the Determination of Residual Formaldehyde by High-Performance Liquid Chromatography" was published in 2022. Journal: Int J Anal Chem.

To the 5.0 mL solutions, 100 *μ*L of the acetic acid solution (200 *μ*g/mL) and 1.0 mL of the MBSH solution (2 mg/mL) were added. A stirring magnet was introduced into the vial and stirred at 500 rpm for 50 minutes for the derivatisation reaction to reach an equilibrium. To an HPLC vial, containing 1 mL of acetonitrile, 1 mL of the derivatised standard or sample solution was added and the vial inverted to ensure thorough mixing before injection onto the HPLC.

### 2.3. Instrumentation and Chromatographic Conditions

High-performance liquid chromatographs with UV detectors (models 1200 and 1260, Agilent Technologies, Santa Clara, California, USA) were employed using an ACE 5 C18 (150 × 4.6 mm, 5 *μ*m) column (Advanced Chromatography Technologies Ltd, Aberdeen, United Kingdom). The column temperature was set at 30°C, and an injection volume of 15 *μ*L and a flow rate of 1.0 mL/min were used. Data were acquired at 193 nm.

The autosampler was uncontrolled at ambient temperature (15–20°C) during the analysis, and an isocratic flow with a run time of 15 minutes was employed using eluent A (premixed 0.07% v/v formic acid in water/acetonitrile: 70/30).

## 3. Method Development, Validation, and Allowable Intake

Different parameters were studied and optimised, such as derivatisation time, detection wavelength, and eluent composition, with the aim to successfully prove solution stability, sensitivity, peak resolution, and carryover.

Subsequently, the developed method was validated according to ICH guideline Q2 (R1) [63]. Selectivity, linearity, limit of quantification, accuracy, precision, intermediate precision, and solution stability were successfully demonstrated.

For the validation of the method, a specification limit needed to be established.

Impurity specification limits are set based upon their allowed daily intake, as specified in the relevant ICH guidelines [6, 7, 64, 65], their fate and purge in the synthesis steps leading to the API and the drug daily intake.

Regarding formaldehyde, permissible limits have been reported in ICH M7(R1) [66], in which the following is stated: “higher acceptable intakes may be justified when human exposure to the impurity will be much greater from other sources, for example, food, or endogenous metabolism (e.g., formaldehyde). For example, formaldehyde is not a carcinogen orally, so that regulatory limits have been based on noncancer endpoints. Health Canada (Ref. 8), WHO IPCS (Ref. 9), and US Environmental Protection Agency (EPA) (Ref. 10) recommend an oral limit of 0.2 mg/kg/day or 10 mg/day for a 50 kg person.” For a 300 mg daily dose of the drug substance, the allowable formaldehyde intake would therefore be about 33,000 *μ*g/g for a 50-kg person. Considering the formaldehyde levels found in research samples (<1000 *μ*g/g), its fate and purge in the compounds of interest, and its allowable intake in pharmaceutical applications, discussed above, a limit of no more than 1000 *μ*g/g was used for the method validation.

The article "Novel Method of Analysis for the Determination of Residual Formaldehyde by High-Performance Liquid Chromatography" was published in 2022. Journal: Int J Anal Chem.

## 4. Results and Discussion

### 4.1. Derivatisation Development and Optimisation

The method herein is based upon a derivatisation reaction between formaldehyde and MBSH, forming the correspondent derivative, which is highly UV active and therefore easily detected by HPLC-UV.

The derivatisation time was optimised by derivatising a 6.0 *μ*g/mL standard solution (corresponding to 1000 *μ*g/g in the material) in duplicate for 0, 10, 20, 35, 50, 65, and 80 minutes (squares, Figure 2), and injecting each solution on the HPLC. The solutions were later re-injected, approximately 240 minutes after the first injection (circles, Figure 2). Recoveries (%) were calculated against the 50 minutes of derivatisation point, and the acceptance criteria range of 90.0–110.0% is represented by the space between the two dashed lines in Figure 2. Results show lower recoveries for the first set of injections, with the first two points (0 and 10 minutes) giving recoveries below 90.0%, compared to those of the re-injections, up to a derivatisation time of 20 minutes. On the contrary, the recoveries for the re-injections were consistent across all times tested. Furthermore, better agreement between the two sets of injections was obtained at 35 and 50 minutes, demonstrating that the derivatisation end point was reached. As it is crucial to reach an equilibrium before the solutions are transferred into vials for analysis, a 50-minute derivatisation was selected; this is lower than times employed by some methods in the literature [12, 14, 48]. If time is a critical factor, lower derivatisation times (30–35 minutes) may be employed, as shown in Figure 2, similarly to other derivatisation methods found in the literature [53, 56, 67]. Standard and sample solution stability was successfully demonstrated when using this derivatisation time, as described in the “Standard and sample stability” section.

The detection wavelength was optimised by selecting the wavelength showing no interferences from any of the eluent or synthesis components and the bigger response and signal top noise ratio within the 193, 230, and 254 nm range, therefore showing higher sensitivity (Figure 3 and Table 1). A maximum absorbance wavelength of 193 nm was selected, which is within the range of the maximum absorbance obtained in several formaldehyde/MBSH derivatisation product UV spectra, where values between 192 nm and 194 nm were observed. An example UV spectrum is shown in Figure 4. In addition to greater sensitivity, no interferences were observed at this wavelength at the retention time of the derivative peak.

The article "Novel Method of Analysis for the Determination of Residual Formaldehyde by High-Performance Liquid Chromatography" was published in 2022. Journal: Int J Anal Chem.

The eluent composition was optimised to a premixed 0.07% v/v formic acid in water/acetonitrile: 70/30 solution, as this combination gave good peak resolution between the derivative peak, the reagent, and sample peaks.

We carryover after the injection of the 6.0 *μ*g/mL standard solution was tested; no peaks at the retention time of the formaldehyde/MBSH derivatisation product could be observed, demonstrating no carryover.

## 5. Method Validation

### 5.1. Selectivity

Selectivity was tested by separate injections of diluent, reagent blank, and a formaldehyde-free sample spiked with the relevant reagents used in the synthesis of the samples under investigation at the optimised wavelength. The method was demonstrated to be selective as no significant interfering peaks (below the quantification limit QL/10) were observed for the formaldehyde/MBSH derivatisation product peak. The method was, therefore, deemed selective. The retention times of MBSH and the derivative peak were 3.2 and 5.2 minutes, respectively (Figure 5).

### 5.2. Sensitivity

As per ICH Q2(R1) [63], an analyte peak with a signal-to-noise ratio of not less than 10 : 1 is considered quantifiable. The QL of this method was set at 83 *μ*g/g (0.5 *μ*g/mL in solution), with this concentration giving a signal-to-noise ratio (S/N) of 88 : 1, calculated following the method shown in USP <621> [68]. Furthermore, at this level, formaldehyde can be quantitatively determined with suitable precision and accuracy in samples. Repeatability and accuracy were demonstrated from six spiked samples at this level (Table 2).

This QL is suitable for a proposed limit for formaldehyde set at 1000 *μ*g/g; however, although it is not a requirement for the purpose of this work, based upon the signal-to-noise ratio at the QL, the method is capable of quantifying lower formaldehyde concentrations than 0.5 *μ*g/mL (corresponding to 83 *μ*g/g in the sample, per method sample concentration), if necessary.

Increasing the sample concentration can also contribute to enhancing the sensitivity further, matching other available methods using different derivatising reagents and detection techniques. This is particularly applicable to aqueous soluble samples, water samples, and sample extraction procedures employing aqueous diluents for more complex matrices.

### 5.3. Linearity

A seven-point calibration of the formaldehyde/MBSH derivatisation product peak was performed (83–2500 *μ*g/g, concentrations in the sample). Each solution was injected onto the HPLC, and the derivative peak integrated from the extracted chromatograms.

The article "Novel Method of Analysis for the Determination of Residual Formaldehyde by High-Performance Liquid Chromatography" was published in 2022. Journal: Int J Anal Chem.

A calibration curve was constructed using unweighted linear regression of the integrated derivative peak area versus the nominal formaldehyde concentrations (see Figure 6).

A correlation coefficient (*R*^2^) of 0.9999 was achieved, demonstrating good linearity between derivative peak area and formaldehyde concentration in the range of 83–2500 *μ*g/g. The obtained correlation coefficient is comparable or greater than values found for other reported methods. Furthermore, the tested range was established based upon the proposed limit of 1,000 *μ*g/g; as explained in the “sensitivity” section, low concentrations could be included for linearity, if needed.

### 5.4. Accuracy (Recovery)

Accuracy was demonstrated by calculating the recovery of formaldehyde in spiked samples at four levels and by calculating standard concordance at the proposed specification limit (1000 *μ*g/g). The four levels correspond to 83 *μ*g/g (QL), 167 *μ*g/g (low), 1000 *μ*g/g (mid), and 1667 *μ*g/g (high).

Three spiked sample replicates were prepared at the low and high levels, and six replicates were prepared at the mid level and at the QL. Recoveries between 70.0 and 130.0% were obtained at the QL, and recoveries between 80.0 and 120.0% were obtained at low, mid, and high levels, for both samples (Table 2). An average recovery of 107.4% was obtained across the four levels, showing high accuracy. This is in line or superior to what was observed for other methods in the literature and what is requested for method validation in the pharmaceutical industry. An example chromatogram overlay of a blank and spiked sample at the limit is presented in Figure 7.

Two formaldehyde standards were prepared at 1000 *μ*g/g; seven replicates from standard 1 were injected followed by 2 injections of standard 2. Standard concordance was calculated between the average of the 7 standard 1 injection and the average of the 2 standard 2 injections, giving a value of 100.3% and consequently indicating good standard accuracy (Table 3).

## 6. Precision

### 6.1. Repeatability

The results obtained for the accuracy tests were used to prove method repeatability. The percentage relative standard deviation (%RSD) was calculated for the spiked samples at the four levels, and values below 5.0% were obtained in all cases (Table 2).

### 6.2. Intermediate Precision

Intermediate precision was demonstrated by successful use of the method by six different analysts, on 33 different days over a period of three years, using four different HPLC systems and three columns with different serial numbers. Furthermore, more than 220 samples were analysed as part of Design of Experiment (DoE) investigations with the aim to optimise the synthesis process of an API (hydromethylthionine mesylate (HMTM), also known as *N,N,N′,N′*-tetramethyl-10*H*-phenothiazine-3,7-diaminium bis(methanesulfonate)) [69–71]. On each occasion, a 6.0 *μ*g/mL (1000 *μ*g/g in the material) standard was prepared in duplicate (1 and 2); standard 1 was injected six times from separate unpierced HPLC vials, followed by an injection of standard 2. System precision and standard concordance were satisfied in all cases. RSD (%) values below 5.0% and standard concordance values between 95.0 and 105.0% were obtained.

The article "Novel Method of Analysis for the Determination of Residual Formaldehyde by High-Performance Liquid Chromatography" was published in 2022. Journal: Int J Anal Chem.

Intermediate precision was also demonstrated during validation of the method at a CMO in the United Kingdom (UK) under good manufacturing practice (GMP) (see “Reproducibility” section).

### 6.3. Reproducibility

Interlaboratory reproducibility was proven by a full validation of the method under GMP at a CMO in the UK, where specificity, repeatability, intermediate precision, accuracy, linearity, limit of detection, limit of quantification, robustness, and solution stability have been proven.

### 6.4. Standard and Sample Stability

The stability of the formaldehyde working solution (6.0 *μ*g/mL), underivatised and stored in the flask at ambient temperature (15‐20°C) with no light protection, was tested at Day 0 and after 1, 5, and 7 days. Its stability was also tested following derivatisation after 1, 2, and 5 days in pierced HPLC vials stored in the autosampler at ambient temperature (15‐20°C) and in unpierced HPLC vials stored in the autosampler at ambient^1^ and refrigerated (2‐8°C) temperatures. The results showed that the underivatised 6.0 *μ*g/mL formaldehyde solution gave consistent results over the test period of 7 days when kept in the flask at ambient temperature (15‐20°C) with no light protection, while the derivatised 6.0 *μ*g/mL formaldehyde solution in HPLC vials was stable for 5 days both when stored in pierced vials in the autosampler at ambient temperature (15‐20°C) and when stored in unpierced vials at ambient1 and refrigerated (2‐8°C) temperatures. Sample stability was determined by injecting (from unpierced HPLC vials) a reference material and a representative MTC sample containing formaldehyde at around the proposed specification limit (1000 *μ*g/g) over a 5-day period, when stored at ambient (15‐20°C) and refrigerated (2‐8°C) temperatures. Samples displayed stability over a maximum of 2 days when kept at ambient temperature (15‐20°C) and 5 days when stored refrigerated (2‐8°C).

### 6.5. Application to Samples

MTC samples synthesised with different paraformaldehyde equivalents and a sample synthesised using a different synthesis process, which does not employ paraformaldehyde altogether, were analysed for formaldehyde content. The paraformaldehyde used depolymerises during the synthesis process and, upon cooling, formaldehyde remains as a monomer in solution due to the water being produced during the reaction. When the final product is isolated, the residual formaldehyde is incorporated within the solid material.

The article "Novel Method of Analysis for the Determination of Residual Formaldehyde by High-Performance Liquid Chromatography" was published in 2022. Journal: Int J Anal Chem.

Table 4 shows formaldehyde results (*μ*g/g) for two samples of the same material: one synthesised using paraformaldehyde and one without.

As it is possible to observe, formaldehyde was detected and quantified in sample 1 (1300 *μ*g/g), whereas formaldehyde below the QL (83 *μ*g/g) was observed in the sample 2, demonstrating that the method is capable to determine formaldehyde if used in the synthesis process.

The formaldehyde content results obtained for samples synthesised using different paraformaldehyde equivalents, as part of DoE investigations, and the respective percent difference from target paraformaldehyde equivalents are presented in Table 5.

The formaldehyde levels observed increase with the amount of paraformaldehyde used, showing that the method can detect excess amounts of paraformaldehyde in DoE samples.

## 7. Conclusions

A novel analytical method for the quantification of formaldehyde in pharmaceuticals has been developed and validated as per ICH Q2(R1) guideline. The proposed method involves the derivatisation of formaldehyde using 4-methylbenzenesulfonohydrazide (MBSH) and the analysis of the corresponding formaldehyde-MBSH derivative by HPLC-UV.

This method was demonstrated to be selective for the accurate and repeatable quantification of formaldehyde in a pharmaceutical, using a readily available technique of analysis in industry (HPLC-UV) and a widely available and safer derivatising reagent for storage and transportation, compared with the most commonly used DNPH. Intermediate precision, reproducibility, and solution stability were also established.

Furthermore, it has been demonstrated that the method is able to determine whether formaldehyde is used in the synthesis process and detect excess amounts of paraformaldehyde in Design of Experiments (DoE) samples. This has been used to optimise the paraformaldehyde equivalents employed during reaction optimisation investigations.

Numerous samples were analysed in support of DoE using this methodology.

The excellent robustness and reproducibility of the proposed method allowed a contract manufacturing organisation (CMO) in the UK to validate the procedure under good manufacturing practice (GMP).

The article "Novel Method of Analysis for the Determination of Residual Formaldehyde by High-Performance Liquid Chromatography" was published in 2022. Journal: Int J Anal Chem.

## Figures and Tables

**Figure 1:** Postulated mechanism of reaction between formaldehyde and 4-methylbenzenesulfonohydrazide (MBSH) under acidic conditions.

**Figure 2:** Recoveries (%) of a 6.0 *μ*g/mL standard solution (corresponding to 1000 *μ*g/g in the material) derivatised for 0, 10, 20, 35, 50, and 80 minutes (squares). The solutions were re-injected after 240 minutes (circles).

**Figure 3:** Formaldehyde standard (83 *μ*g/g) chromatograms at different detection wavelengths (193 nm in green, 230 nm in blue, and 254 nm in black), showing the formaldehyde/MBSH derivative peak.

**Figure 4:** UV spectrum of the MBSH/formaldehyde derivative peak.

**Figure 5:** Diluent (dashed line), reagent blank (dotted line), and formaldehyde standard (solid line) chromatograms showing the retention time of 4-methylbenzenesulfonohydrazide (MBSH) and the formaldehyde/MBSH derivative peak.

**Figure 6:** Derivative peak calibration; signal area (mAU × second) of the formaldehyde/MBSH derivative plotted against the formaldehyde concentration in the sample (*μ*g/g).

**Figure 7:** Blank (black line) and spiked sample (blue line) chromatograms at the proposed limit of 1000 *μ*g/g, showing the retention time of 4-methylbenzenesulfonohydrazide (MBSH), the formaldehyde/MBSH derivative, and sample peaks.

**Table 1:** Formaldehyde/MBSH derivative signal-to-noise ratios for a 83 *μ*g/g formaldehyde standard at 193, 230, and 254 nm.

	Signal-to-noise ratio		
Formaldehyde concentration (*μ*g/g)	193 nm	230 nm	254 nm
83	88:1	82:1	72:1

**Table 2:** Spiked sample recoveries (%) and RSD (%) at QL, low, mid, and high levels.

Spiked samples	Recovery (%)	RSD (%)
QL A	114.1	3.3
QL B	115.0	
QL C	108.4	
QL D	119.2	
QL E	111.7	
QL F	110.9	
Low spike A	101.8	1.9
Low spike B	105.4	
Low spike C	105.1	
Mid spike A	105.5	0.4
Mid spike B	104.7	
Mid spike C	104.7	
Mid spike D	105.3	
Mid spike E	105.0	
Mid spike F	105.7	
High spike A	103.4	0.3
High spike B	103.9	
High spike C	103.4	

**Table 3:** Peak areas (mAU *x* second) of two 1000 *μ*g/g formaldehyde standards (seven injections of standard 1 and two injections of standard 2) and the concordance (%) result.

	Area (mAU *x* second)
Standard 1 A	2220.91
Standard 1 B	2233.58
Standard 1 C	2236.76
Standard 1 D	2215.49
Standard 1 E	2227.64
Standard 1 F	2242.16
Standard 1 G	2232.05
Average standard 1	2229.80
Standard 2 A	2244.25
Standard 2 B	2228.95
Average standard 2	2236.60
Concordance (%)	100.3

**Table 4:** Formaldehyde content (*μ*g/g) for two samples, one synthesised using paraformaldehyde and one without.

Sample	1	2
Paraformaldehyde used in synthesis	Yes	No
Formaldehyde content, *μ*g/g	1300	<QL (83 *μ*g/g)

The article "Novel Method of Analysis for the Determination of Residual Formaldehyde by High-Performance Liquid Chromatography" was published in 2022. Journal: Int J Anal Chem.

**Table 5:** Formaldehyde content (*μ*g/g) and respective difference (%) from target paraformaldehyde equivalents used as a part of the synthesis process.

Sample	3	4	5	6
Paraformaldehyde, % difference from target equivalents	−2.0	−1.0	+1.0	+2.0
Formaldehyde content, *μ*g/g	708	1130	1456	1565

## Data Availability

The data used to support the findings of this study are included within the article.
